# Recognition of Handwritten Medical Prescription Using Signature Verification Techniques

**DOI:** 10.1155/2022/9297548

**Published:** 2022-09-17

**Authors:** Seerat Rani, Abd Ur Rehman, Beenish Yousaf, Hafiz Tayyab Rauf, Emad Abouel Nasr, Seifedine Kadry

**Affiliations:** ^1^Department of Computer Science, University of Gujrat, Gujrat, Pakistan; ^2^Centre for Smart Systems, AI and Cybersecurity, Staffordshire University, Stoke-on-Trent ST4 2DE, UK; ^3^Industrial Engineering Department, College of Engineering, King Saud University, Riyadh 11421, Saudi Arabia; ^4^Department of Applied Data Science, Noroff University College, Kristiansand, Norway; ^5^Department of Electrical and Computer Engineering, Lebanese American University, Byblos, Lebanon

## Abstract

Patient record keeping plays a vital role in diagnoses and cures. Due to a shortage of time, most doctors write prescriptions manually in Pakistan. At times, it becomes difficult for pharmacists to read prescriptions properly. As a result, they may dispense the wrong medicine. This might cause risky and deadly effects on the patient's health. This paper proposes an online handwritten medical prescription recognition system that lets doctors write prescriptions on a tablet using a stylus and automatically recognizes the medicine. We use signature verification techniques to recognize the doctor's handwriting to overcome the problem of misinterpretation of the medicine name by the pharmacist. The proposed system stores different features like the pen coordinates, time, and several pen-ups and pen-downs. Besides using features already proposed in the literature for signature verification, we propose some new features that greatly enhance recognition accuracy. We built a dataset of 24 medicine names from two users and compared results using newly proposed features. We have obtained 84%, 78%, 77.47% 77.31%, 74.17%, 60%, 38.5%, 68%, and 61.64% accuracies for 9 users using SVM classifier.

## 1. Introduction

Computers are used in almost every domain of daily life, like businesses, industries, entertainment, education, personal management, and research activities. Data can be processed and reproduced in a speedy way using computers. Patient record management helps practitioners to diagnose and continue the care timely. Computerized patient record management systems are used to maintain the record of patients and employees working in the hospital [1, 2]. Health care is a broad area that deals with health care information, medical device information, pharmaceutical information, hospital management, and biological system. In the health care system, patient's precaution and patient care are the major goals [3, 4].

In developing countries like Pakistan, most hospitals, especially in the public sector, are not computerized. Due to a high patient-to-doctor ratio, doctors have a hectic schedule where they have to prescribe or take notes while standing or in walking conditions in emergency cases. Handwritten prescriptions are widely used in the tropical areas of mid-Asia. Especially in Pakistan, doctors mostly prefer to write handwritten prescriptions because they feel comfortable writing the prescription manually, even if they have enough time to access and use a computer.

Handwritten prescriptions have several potential threats associated with them. Unreadable handwriting prescription and the incapability of pharmacists to understand medicine names in medical prescriptions are causing a notable number of patients to expire [5]. Patients may get delayed or wrong medical dosage due to wrong interpretation of handwritten prescription, which may result in further severity of disease and even patient's death.

Biometric verification is employed in several real-life business applications. It provides numerous benefits like it is difficult to be stolen, hacked, and forged. Biometrics deals with bioscience, which means the automatic identification of a human's physiological or behavioral characteristics. The biometric method is preferred over passwords and PINs for easiness of use, accuracy, and case sensitivity. There are different biometric types, such as fingerprint, iris, and face recognition [6].

Biometrics can be found in an extensive range of applications which include physical access control systems, logical access control services, consumer identification, prescription identification, and authentication. Handwritten signature verification is still widely used techniques. The biometric system performs two tasks: verification and identification [7].

The signature verification system is intended to verify the individuality of a person by recognizing their handwritten signature. Signature verification contains two types online and offline signature verification [8]. Offline techniques capture image of the signature after the person has completed writing. Online signature verification techniques capture feature which person is signing. It is done by using a tablet and stylus and recording features pen coordinates, time, pressure, etc. Signature verification includes three basic steps [9–12]. The first step is preprocessing and contains the data in raw form. After preprocessing, the features from obtained data are extracted in numeric form. In the third step, the classifier obtains results and checks whether the signatures are genuine or forged. There are many classifiers, such as neural network (NN), support vector machine (SVM), nearest neighbor, hidden Markov model (HMM), time delay neural networks, and Naive Bayes, which have been employed for signature verification [9]. Several studies in the related work are found on the optimization algorithm that can be used to solve machine learning healthcare-related optimization problems, such as the Bat algorithm [13] and particle swarm optimization [14].

For effective results, features should be dense enough and provide a better understanding of signatures because it is considered personal identification [15, 16]. In [8] offline recognition system, they used a static representation of documents to take a signature on paper which is later scanned which includes cheque, form, and documentation authentication. Offline signature verification techniques are famous for limited information [15]. Offline processing is also a difficult task due to the deficiency of dynamic characteristics [17].

On the other hand, an online recognition system uses dynamic representation, in which information can be stored at runtime. Electronic tablets [18, 19] and smartphones have on-line recognition writing interface [8, 20–22]. Most applications are based online, where a person acts and the system automatically derives data for authentication. Online verification is stronger than the other approach because it provides a higher level of security and stores dynamic features such as pressure, coordinates, pens up, and pens down. Online signature verification can be divided into two types:

- The parametric approach is used to extract the features from signals such as speed, pressure, coordinates, and the number of the pen up and pen down
- The functional approach is used for analyzing the online signatures

The representation of offline verification is shown in Figure 1.

The contribution of this work is as follows:

- We propose an online medical prescription recognition system to overcome problems of unreadable handwriting prescription
- We use signature verification techniques to recognize the medicine name prescribed by a doctor
- We use tablet and stylus, like used in [23, 24], to enable doctors to prescribe in the same way they normally do

## 2. Literature Review

### 2.1. Signature Verification

Signature verification is a broad area in biometric. It has been considered an essential component of the study conducted by the researchers due to the extensively utilized signature verification techniques for experimentation.

In [25], the author proposed a secure retrieval of the classified information system using the neuro-fuzzy technique. The neuro-fuzzy technique was based on a fuzzy neural network. Dynamic signatures were tested by using Svc 2004 database. They extracted different features, including total time duration, average pen pressure, and dynamic pen pressure. The verification system was suitable; the obtained EER of the overall system was 3.952%. The proposed scheme was beneficial for the practical application of classified information.

Online signature verification uses effective and simple techniques. In their research [26], the author employed two types of features, the first was based on the histogram, and the second was based on quantized features using a model-free Manhattan distance classifier. Several tests were conducted on MCYT and SUSIG datasets. The obtained results of the proposed technique were similar to state-of-art algorithms despite their simplicity and efficiency.

The author reviewed the signature verification system, which included feature extraction algorithms [27], tablet PC, digitized pen, HMM's, modified dynamic time warping technique (DTW), and NN techniques and methodologies.

They discussed the main challenges of signature verification: signature inconsistency and intraperson variability. Different steps performed for signature verification included signature acquisition, preprocessing, feature extraction, threshold selection enrolment, and matching. The steps performed in preprocessing were smoothing, normalization, and segmentation.

In the feature extraction step, performance evaluation parameters were involved, which derived false acceptance rate and false reject rate. The obtained results of the false acceptance rate (FAR) were 0.25%, and the false reject rate (FRR) was 0.5%.

In [28], the study is carried out to propose both online and offline verification approaches. The webcam was used for data collection, preprocessing, and feature extraction, including pen up and pen down, and then, classification results were obtained based on online verification. However, for offline verification, they collected data through the image, performed preprocessing and feature extraction, and in the end, obtained results from different classifiers. When those steps were completed on both online and offline approaches, then these were combined and used SVM for final verification.

Discrete cosine transformed (DCT) and sparse representation techniques [29] are used for signature verification and discussed new properties of DCT, including time-series and extracting different energy features (*x*, *y* coordinate, pressure, azimuth, and altitude). For experimental evaluation, they used SUSIG-visual and SVC2004 databases. In the end, the obtained error rate was 0.33%.

In 2016, the author [15] proposed a two-stage classification approach combining generative and discriminative modeling principles for online handwritten character recognition. The first stage was based on HMM and presented a few unknown patterns in candidate characters. HMM returned the top-ranking character out of the total number of classes. In the second stage, they used SVM frequency count analysis and chose one character from the candidate character class.

The frequency count analysis was used for pairwise classifiers and same-shape characters. The two-stage approach was better than the single-stage.

In [30], they used handwritten signature verification techniques to propose hand-worn devices for genuine and forged signatures. Sixty-six applicants were included in this experiment. Data were collected in two stages; the major one was participants providing genuine signatures, and the second was forged signatures. They collected three types of datasets from accelerometer and gyroscope, which included the acceleration of accelerometer, angle of acceleration, and angle of velocity. This method provided 0.98 AUC and 0.05 EER high degree of accuracy amongst genuine and forged signatures.

In [31], the author introduced handwriting recognition techniques for Chinese characters conVent (conventional neural network) and direct Map (direction decomposition). Direct Map and conVent provided better efficiency and accuracy than the other techniques. These techniques reduced the mismatch problem between the train and tested the data. The ConVent was interesting and straightforward for the recognition system.

In [32], the authors carried out the NN model for signature verification using autoassociative memory. NN model reads the image of signature in the form of matrices. In [33], an automatic signature recognition approach was introduced. Gabor filter techniques were used for preprocessing signature images and then performed linear discriminant analysis. After that, they applied NNs used for matching the trained data. If the data matched to original data, then making a decision data is authentic or inauthentic. The obtained results from the proposed system were very high, 99.5%, rejection rate of 73%, and computational time of method were 0.87 s.

### 2.2. Prescription Recognition

The authors [5] used MediPic and Android applications to resolve the recognition problem. They used optical character recognition technology to scan the medicine name and convert it into a digital script. They used Tesseract for character recognition and an inner key algorithm to match the characters. The inner key algorithm matched the character and returned the best results in the database. The MediPic provided more efficient results and helped to decrease the misunderstanding of medicine names.

In [34], the author presented a design of printed traditional Chinese medicine (TCM) prescription and filing system based on the Microsoft office document imaging (MODI) and optical character recognition (OCR) engine.

An optical recognition engine [35] extracted complete information about the disease and stored the data in the database and made a file for further use. TCM provides information for future use. In 2017, [36] implemented a hospital information management system for medical records. Using fingerprints of patients for authentication because health is the main aim or goal of the hospital.

In addition to the health of patients in hospitals, their privacy and security are also considered. They used different technologies for biometric authentication, which included data management, system design, unified modelling language, biometrics, and computer programming. The efficiency of the hospital was increased by using a medical record system with biometric authentication.

In [37], handwritten medical prescription systems were introduced; a prescription is written by doctors based on word spotting and uses an information retrieval approach. They proposed two approaches: the first was Tandem-HMM, used for word spotting, and the second was domain knowledge, used to reduce the text information, which increased the performance.

Different steps were involved: the first one was developing a diagnostic system. The second was information extraction, the third was wrong medication detection, and the fourth was a statistical analysis of medical prescriptions prescribed by doctors. The obtained accuracy was increased by 15.42%, which was a good achievement.

Different techniques are used for medical prescription recognition problems, but our focus is to use signature verification techniques for medical prescriptions. A summary table concerning different coordinates is presented in Table 1.

## 3. Methodology

Patients' death due to the wrong drug intake caused by misinterpreted prescriptions by pharmacists happens frequently. Most doctors write prescriptions manually because prescribing a stylus on a tablet is not very common or practiced regularly in Pakistan for prescription writing. Therefore, sometimes, it causes harmful effects on patients. Our work is based on handwritten medical prescriptions, but we employed signature verification techniques.

### 3.1. Signature Verification vs. Handwritten Medical Prescription

- Through the signature verification technique, we can verify a person's identity by recognizing their handwritten signature. Signature verification uses a pattern matching technique to verify the signatures, but most of the time, it is difficult to read the signature because there is no pen up and pen down movement Signatures can be forged easily. Offline signature verification is only based on shapes
- Through the handwritten medical prescription, the doctor's handwriting is recognizable. The forgeries or forged signatures are automatically involved in the signature verification. Forged signatures are referenced or duplicate signatures of a person. Online handwritten medical prescription recognition is based on character recognition. Pen up and pen down are associated with handwritten medical prescriptions. There are two types of handwritten verification techniques called online and offline verification. Both techniques are linked with signature verification and handwritten medical prescription recognition

### 3.2. Offline and Online Handwritten Verification

- The offline technique deals with the only shape of the writing and is used for limited information due to its static representation of documents to take a signature or prescription on paper. This prescription is later scanned. This approach is difficult because the segmentation is performed on scanned data. Through the offline approach, we cannot calculate the speed and pressure of a pen
- Compared to the offline technique, the online approach is more secure and accurate due to the variation of feature value each time and provides relevant results. The online approach deals with dynamic features such as speed, pen up, pen down, and pressure. A tablet or smartphone is used for an online approach that stores the pen tip movements as well as pen up and pens down, switching

In this article, we have proposed signature verification techniques for medical prescription recognition systems to overcome the misinterpretation of medicine names. There are five steps involved in medical prescription recognition explained below:

- In the phase of data acquisition, we collected data from two users and 9 users, and we used the stylus for writing a medicine's name on the tablet, which stores the movements of the stylus
- Feature extraction is the second step. We extracted different features from the original data obtained from the medical prescription system. Several extracted features involved: pen up with respect to *x*-*y* coordinates, pen down with respect to x-y coordinates, the total time between pen down to pen up, midpoints of total time with respect to *x*-*y* coordinates, quarter midpoints of total time with respect to *x*-*y* coordinates, and three-quarter of total time with respect to *x*, *y* coordinates
- Preprocessing is the third step in which the unwanted data have been removed, i.e., useless columns or extra columns and adding missing values
- We have carried out different classifiers for the experimental evaluation, which involves Naive Bayes, SVM, gradient boosted, and decision tree.  Figure 2 presents a flow of the complete research activity

### 3.3. Data Acquisition

Data acquisition is a process that measures the physical condition and converts it into digital numeric values. The doctor prescribes the tablet using a stylus. Our proposed system calculates the movement of a stylus according to *x* and *y* coordinates.

Medicine name has already been stored in the database of the proposed system. The user has to put the medicine name by using the styles into the GUI interface of the proposed system. After that, system generates values according to pen movement in the form of *x* and *y* coordinates. The system generates an event that includes the number of *x*-coordinates, *y*-coordinates, total time, and pens up, and pens down. The real-time data experiment of the proposed system is presented in Figures 3 and 4.

Original data obtained from the proposed medical prescription application is given in Table 2.

### 3.4. Feature Extraction

We extracted the features from the acquired data. When the medicine name is written on the GUI of the proposed system, then the original number of strokes or movements of the stylus are recorded and accumulated in the database. We extracted two types of features called spatial and local spatial features.

#### 3.4.1. Spatial Features

Spatial features are also called static features which are extracted from the shape of the signature or original. The extracted spatial feature is shown in Table 3.

#### 3.4.2. Local Spatial Features

Local spatial features are extracted for signature verification which includes: *x*, *y* coordinates, total time, pen up, pen down, and angle.

Apart from the spatial features, we have extracted different features, including the following:

- Pen down with respect to the *X* coordinate (dnx): the system calculates values according to the *x* coordinate as soon as the stylus touches the screen of the tablet
- Pen down with respect to the *Y* coordinate (dny): the system calculates values according to the *y* coordinate as soon as the stylus touches the screen of the tablet
- Pen up with respect to *X* coordinate (upx): the system calculates values according to the *x* coordinate when the user takes a pause or lifts the pen for the first time while writing
- Pen up with respect to the *Y* coordinate (upy): the system calculates values according to the *y* coordinate when the user takes a pause or lifts the pen for the first time while writing

(v) Total time of pen up (time): the total time of pen up is the total time of lifting the pen from the tablet by the user according to coordinates

- Midpoints of pen up with respect to the *X* coordinate(midpoints *x*): pen up midpoints are middle points of the total time of pen up from the tablet with respect to the *x* coordinate or the total time between pen up and pen down
- Midpoints of pen up with respect to the *Y* coordinate (midpoints *y*): midpoints are middle points of the total time of pen lifting from the tablet with respect to the *y* coordinate. Or the total time between pen up and pen down
- Quartiles of pen up with respect to *X* coordinate (quarter *x*): quartiles of pen up are the first total time divided into four equal parts with respect to the *x* coordinate
- Quartiles of pen up with respect to *Y* coordinate (quarter *y*): quartiles of pen up are the total time divided into four equal parts with respect to the *y* coordinate
- Third quartile midpoints of pen up with respect to *X* coordinate (3quarter *x*): third quartile pen up midpoints are the three equal parts out of one-quarter of total time with respect to the *x* coordinate
- Third quartile midpoints of pen up with respect to *Y* coordinate (3quarter *x*): third quartile pen up midpoints are the three equal parts out of one-quarter of total time with respect to the *y* coordinate

The accuracy obtained by using the feature includes upx1, upy1, dnx1, dny1, time1, midpoints1x, midpoints1y, quarter1x, quarter1y, 3quarter1x, and 3quarter1y with SVM was not high enough. To boost the accuracy, we extracted some additional features, including total time, midpoints of total time, quarter time of midpoints, and 3quarter time of midpoints. We used a six-time pen up and pen down, as shown in Table 4.

### 3.5. Preprocessing

There exist some irrelevant data obtained from feature extraction which cannot be used in its original form. It contained useless content such as the first pen down *x* column, the first pen down *y* column, and attributes containing missing values and extra columns. This type of data has not been used in our experiments. We have cleaned up (error-free) the irrelevant data to get the best results.

#### 3.5.1. Remove Columns

Two columns are considered useless because the first pen down concerning the *x*-coordinate and the first pen down concerning the *y*-coordinate contain “0” values. These columns have been removed. Furthermore, we took only six times to pen up and pen down, so extra columns are removed as unnecessary. This data does not affect the analysis. The description of data that is removed is given in Table 5.

### 3.6. Missing Values

Several attributes of the columns contain null values during writing medicine names. The null values affected the result analysis because the classifier does not accept these types of data and shows an error to add values containing null values. Therefore, to improve the results, we replaced “0” with the null attribute in Table 6.

### 3.7. Dataset

We collected data for 100 medicine from 2 users while data for 24 medicine from nine users. Each medicine contains at least 10 samples for the training dataset. The total number of training data is 3000 medicine samples. Each sample is labeled with its respective medicine name. The user name is also included to train the classifier for each user separately. The sample of training data is shown in Table 7.

The classifier employed in this work is given the same features as input, the same classes of medicine, and the same number of medicines. We used the KNIME analytics platform for analysis. It is an open-source platform to verify the online signature (medicine name) of samples.

#### 3.7.1. *F*-Measures

We have measured the performance of eleven features, including pen up *x*, pen up *y*, pen down *x*, pen down *y*, total time, midpoint *x*, midpoint *y*, quarter *x*, quarter *y*, 3quarter *x*, and 3quarter *y*, with different classifiers. Features are ranked using all the eleven feature ranking metrics. The performance of feature ranking metrics is compared with different classifiers. Macroaverage *F*1 and microaverage *F*1 are used to calculate classification performance. Precision and recall are the harmonic means of *F*1-measure. Description of macro-*F*1-measure is given below.

(1) $$\begin{array}{c} \text{Macro Average }F1=\overset{C}{\underset{k=1}{\sum }}\frac{\left(2\times P_{k}\times r_{k}\right)/\left(P_{k}+r_{k}\right)}{C}, \end{array}$$

where *p*_*k*_ is the precision and *r*_*k*_ is the recall values of class *k*. Furthermore, it sums up the global precision and recalls for all classes of the dataset in the micro-*F*1 measure as given below.

(2) $$\begin{array}{c} \text{Micro Average }F1=\frac{2\times P\times r}{P+r}, \end{array}$$

where *p* is the precision and *r* is the recall which is dependent on the overall performance of the classification decisions within the entire dataset.

(3) $$\begin{array}{c} \text{Precision}=\frac{\text{tp}}{\text{tp}+\text{fP}},\\ \text{Recall}=\frac{\text{tp}}{\text{tp}+\text{fn}}, \end{array}$$

where tp is the true positive value, fp is the false positive, and fn is the false negative value, respectively.

## 4. Results and Discussion

The accuracy obtained using this chunk of the dataset is 90% using SVM, as compared to Naive Bayes 70%, gradient boosted 50%, and 40% from the decision tree. The experimental results reveal that SVM outperformed other states of the art algorithms for this experimentation. Empirical results of the pen up and pen down features are obtained from user 1 and user 2; data are shown in Figure 5.

The comparison evaluation on the features: upx1, upy1, dnx1, dny1, time1, midpoints1x, midpoints1y, quarter1x, quarter1y, 3quarter1x, and 3quarter1y have been carried out. In this experimental setup, we used 24 medicine data and achieved 90% with SVM, 75% Naive Bayes, 70% gradient boosted, and 85% decision tree. The accuracy comparison of 20 medicine with 100 medicines for two users is shown in Figure 6. The accuracy can be enhanced if we consider more pen up and pen down features.

We observed that the sample size of the medicine is directly proportional to the accuracy. The more the sample size of medicines increases, the better the accuracy was obtained. The experimental results of classifiers obtained from user 1 and user 9 are shown in Table 8.

We can see from Table 8 that SVM performed better for every user from user 1 to user 9 with higher accuracy of 84% and 78%, 77.47%, 77.31%, 74.1%, and so on. Some users have shown low accuracy because of the slow writing of the medicine name because the time difference of the pen up and pen down was high, which is the reason for less accuracy.

We have computed the *F*1 score, which is the measurement of the test's accuracy defining the weighted harmonic mean of the precision and recall of the test data of all the 9 users.  Table 9 presents the performance of each classifier for *F*-measure obtained data from user 1 to user 9.

The first column of the table shows all the users, and the rest columns confers the *F*-measure of all 9 users' data obtained according to from SVM, Naive Bayes, decision tree, and gradient boosted. The graphical representation of empirical results is shown in Figure 7.

### 4.1. Comparison with Other Features

Through our medical prescription features, we obtained better accuracy; however, additional features can be extracted from original data as described in [41], certain features have been extracted from the handwritten medical prescription application, and the accuracy has been calculated. The proposed features are discussed:

- Pen length (PL): the path length is the total length covered by the user's pen tip throughout the signature creation
- Pen diagonal length (DL): diagonal length is the maximum (*x*max, *y*max) and minimum (*x*min, *y*min) points in the *X*-*Y* coordinate
- Time length (TL): the total time of writing the complete signature (the time period between the first pen down and last pen up)
- Mean speed (MS): mean speed is the average speed and velocity of the user writing the signature
- Covariance *X*-*Y* (CXY): covariance means to measure the scattered points on the signature path
- Vector length ratio (VLR): calculate all vector points of the signatures from the beginning to each *x*-*y* coordinate

We employed the same classifiers with additional features described above obtained from user 1 to user 9 for signature verification. The results of individual classifiers are shown in Table 10.

The comparison of both types of features obtained from user 1 and user 9 is shown in Figures 8 and 9, which infers that the SVM is not proven as a better choice for signature verification features [41].

Furthermore, the overall performance of each classifier is appeared as lower than the proposed prescription recognition system. Further, the observation is recorded that the proposed prescription recognition system was employing signature verification techniques performed better than the others. This confirmed that the local spatial features (extracted features) depend on spatial features (original features).

We obtained significant results from both signature verification features and handwritten prescription recognition systems. The line curves from Figures 8 and 9 show that the overall performance of each classifier remains lower as compared to the proposed handwritten medical prescription recognition system.

## 5. Conclusion

Patients face difficulties when reading doctor-prescribed medication names. This research focused on the performance and analysis of various classifiers for the newly established handwritten recognition system of medical prescription. We used signature verification techniques to recognize the misinterpreted medical prescription issue better. For the performance evaluation of the proposed system, we introduced new features to increase the performance of the prescription system. We achieved 84%, 59%, 57%, and 56% with SVM, Naive Bayes, decision tree, and gradient boosted. Furthermore, the experiment is extended to determine the *F*-measure with 84%, 62%, 59%, and 51% from SVM, Naive Bayes, decision tree, and gradient boosted, respectively. The experimental results revealed that the proposed system based on the handwritten medical prescription data outperformed in terms of better recognition accuracy. This research would help to recognize the prescription in a better way in the area of health care. In the future, we are intended to extract additional features based on statistics. The proposed handwritten medical prescription recognition system opens a new direction for medical prescription recognition.

## Figures and Tables

**Figure 1:** Off-line data representation.

**Figure 2:** Complete research design.

**Figure 3:** Enter medicine name.

**Figure 4:** Write medicine name using stylus.

**Figure 5:** Pen up and pen down features accuracy of user 1 and user 2 data.

**Figure 6:** Comparison of 20 medicine with 100 medicine data.

**Figure 7:** Graphical representation of *F*1-measure score obtained from user 1 and user 2.

**Figure 8:** Comparison of prescription recognition system and proposed signature verification [41] feature data obtained from user 1.

**Figure 9:** Comparison of prescription recognition system and proposed signature verification [41] feature data obtained from user 2.

**Table 1:** Summary table of literature review.

	Features					
Referenced paper	Upx	Upy	Dnx	Dny	Time	Midpoints
[38]	Yes	Yes	Yes	Yes	Yes	No
[39]	Yes	Yes	Yes	Yes	No	No
[40]	Yes	Yes	No	No	No	No
[41]	Yes	Yes	No	No	Yes	No

**Table 2:** Original data obtained from medical prescription application.

Prescription name		Accupril				
Event number	*X*	*Y*	Time from previous	Total time	Up	Down
1	389.552	238.7	0	0	False	True
2	389.552	238.7	3	3	False	False
3	390.593	237.6	31	35	False	False
4	390.802	234.3	5	41	False	False
5	389.864	227.7	14	55	False	False
6	386.427	220.3	17	72	False	False
7	376.532	214.7	17	90	False	False
8	367.678	217.4	16	107	False	False
9	357.783	226	17	124	False	False
10	349.138	239.5	19	143	False	False
11	341.431	262.4	15	159	False	False
12	341.326	275.3	16	176	False	False
13	346.743	283.8	17	193	False	False
14	361.429	285.7	17	210	False	False
15	372.574	278.4	17	228	False	False
16	381.636	265.9	17	245	False	False
17	390.072	243.4	17	262	False	False
18	392.989	234.4	17	279	False	False
19	394.135	232.3	17	296	False	False
20	395.176	232.4	17	314	False	False
21	399.134	238	17	331	False	False
22	403.092	243.7	17	348	False	False
23	408.613	250.9	17	365	False	False
24	420.174	263.4	17	383	False	False
25	428.819	269.4	16	400	False	False
26	439.339	272.6	17	417	False	False
27	448.714	271.8	11	429	False	False
28	448.714	271.8	1	430	True	False
29	494.335	216	111	542	False	True

**Table 3:** Spatial feature obtained from system.

Feature	Description
Upx	Pen up *x*-coordinate
Upy	Pen up *y*-coordinate
Dnx	Pen down *x*-coordinate
Dny	Pen down *y*-coordinate
Time from	Start time of writing
Total time	Total time of complete signature

**Table 4:** Extracted features from original data.

Features	Description
Upx1	First pen up with respect to *x*-coordinate
Upy1	First pen up with respect to *y*-coordinate
Time1	Total time of first pen up
Midpoints1x	Midpoint of first time pen up with respect to *x*-coordinate
Midpoints1y	Midpoint of first time pen up with respect to *y*-coordinate
Quarter1x	Quarter time of the first midpoint pen up with respect to *x*-coordinate
Quarter1y	Quarter time of first midpoint pen up with respect to *y*-coordinate
3quarter1x	3quarter of first midpoint pen up time with respect to *x*-coordinate
3quarter1y	3quarter of first midpoint pen up time with respect to *y*-coordinate
Dnx2	Second pen down with respect to *x*-coordinate
Dny2	Second pen down with respect to *y*-coordinate
Upx2	Second pen up with respect to *x*-coordinate
Upy2	Second pen up with respect to *y*-coordinate
Time2	Total time of second pen up
Midpoints2x	Midpoint of second time, pen up with respect to *x*-coordinate
Midpoints2y	Midpoint of second time pen up with respect to *y*-coordinate
Quarter2x	Quarter time of second midpoint pen up with respect to *x*-coordinate
Quarter2y	Quarter time of second midpoint pen up with respect to *y*-coordinate
3quarter2x	3quarter of second midpoint pen up time with respect to *x*-coordinate
3quarter2y	3quarter of second midpoint pen up time with respect to *y*-coordinate
Dnx3	Third pen down with respect to *x*-coordinate
Dny3	Third pen down with respect to *y*-coordinate
Upx3	Third pen up with respect to *x*-coordinate
Upy3	Third pen up with respect to *y*-coordinate
Time3	Total time of third pen up
Midpoints3x	Midpoint of third time pen up with respect to *x*-coordinate
Midpoints3y	Midpoint of third time pen up with respect to *y*-coordinate
Quarter3x	Quarter time of third midpoint pen up with respect to *x*-coordinate
Quarter3y	Quarter time of third midpoint pen up with respect to *y*-coordinate
3quarter3x	3quarter of third midpoint pen up time with respect to *x*-coordinate
3quarter3y	3quarter of third midpoint pen up time with respect to *y*-coordinate
Dnx4	Fourth pen down with respect to *x*-coordinate
Dny4	Fourth pen down with respect to *y*-coordinate
Upx4	Fourth pen up with respect to *x*-coordinate
Upy4	Fourth pen up with respect to *y*-coordinate
Time4	Total time of fourth pen up
Midpoints4x	Midpoint of fourth time pen up with respect to *x*-coordinate
Midpoints4y	Midpoint of fourth time pen up with respect to *y*-coordinate
Quarter4x	Quarter time of fourth midpoint pen up with respect to *x*-coordinate
Quarter4y	Quarter time of fourth midpoint pen up with respect to *y*-coordinate
3quarter4x	3quarter of fourth midpoint pen up time with respect to *x*-coordinate
3quarter4y	3quarter of fourth midpoint pen up time with respect to *y*-coordinate
Dnx5	Fifth pen down with respect to *x*-coordinate
Dny5	Fifth pen down with respect to *y*-coordinate
Upx5	Fifth pen up with respect to *x*-coordinate
Upy5	Fifth pen up with respect to *y*-coordinate
Time5	Total time of fifth pen up
Midpoints5x	Midpoint of fifth time pen up with respect to *x*-coordinate
Midpoints5y	Midpoint of fifth time pen up with respect to *y*-coordinate
Quarter5x	Quarter time of fifth midpoint pen up with respect to *x*-coordinate
Quarter5y	Quarter time of fifth midpoint pen up with respect to *y*-coordinate
3quarter5x	3quarter of fifth midpoint pen up time with respect to *x*-coordinate
3quarter5y	3quarter of fifth midpoint pen up time with respect to *y*-coordinate
Dnx6	Sixth pen down with respect to *x*-coordinate
Dny6	Sixth pen down with respect to *y*-coordinate
Upx6	Sixth pen up with respect to *x*-coordinate
Upy6	Sixth pen up with respect to *y*-coordinate
Time6	Total time of sixth pen up
Midpoints6x	Midpoint of sixth time pen up with respect to *x*-coordinate
Midpoints6y	Midpoint of sixth time pen up with respect to *y*-coordinate
Quarter6x	Quarter time of sixth midpoint pen up with respect to *x*-coordinate
Quarter6y	Quarter time of sixth midpoint pen up with respect to *y*-coordinate
3quarter6x	3quarter of sixth midpoint pen up time with respect to *x*-coordinate
3quarter6y	3quarter of sixth midpoint pen up time with respect to *y*-coordinate

**Table 5:** Sample cleaning of useless columns.

Medicine	Dnx1	Dny1	Upx1	Upy1
Accupril	0	0	59.16186	33.01608
Accupril	0	0	67.91113	54.263
Accupril	0	0	67.49451	86.75827
Accupril	0	0	49.371	30.72473
Accupril	0	0	-26.0396	66.55288
Accupril	0	0	77.80618	75.82236
Accupril	0	0	76.45212	44.68106
Accupril	0	0	41.66328	47.18067
Accupril	0	0	83.43072	56.55428
Accupril	0	0	46.45455	47.18066

**Table 6:** Sample addition of missing values.

Medicine	Dnx6	Dny6
Accupril	502.355	-21.4552
Accupril	521.5201	0
Accupril	366.2202	-28.0168
Accupril	377.9901	-35.3074
Accupril	0	-50.0969
Accupril	0	21.24692
Accupril	386.1144	-15.5186
Accupril	173.2151	0
Accupril	442.0474	0

**Table 7:** Sample of training data.

Medicine	Upx1	Upy1	Time1	Midpoint1x	Midpoint1y	Quarter1x	Quarter1y
Accupril	59.16186	33.01608	430	372.5739	278.4178	389.5516	238.736
Accupril	67.91113	54.263	356	280.2897	240.819	277.165	214.1562
Accupril	67.49451	86.75827	302	378.3026	217.4891	356.3252	195.8256
Accupril	49.371	30.72473	409	352.3672	264.2531	382.2606	245.2976
Accupril	-26.0396	66.55288	110	328.3066	249.2553	367.9909	213.6355
Accupril	77.80618	75.82236	363	406.3211	181.5568	373.0946	167.9129
Accupril	76.45212	44.68106	356	403.7172	199.9916	379.5525	204.9909
Accupril	41.66328	47.18067	281	280.498	274.9808	312.1621	189.6806
Accupril	83.43072	56.55428	341	372.1572	225.9254	329.2441	212.6981
Accupril	46.45455	47.18066	345	302.4754	211.24	301.2255	200.929

**Table 8:** Accuracy obtained by comparing SVM, Naive Bayes, decision tree, and gradient boosted on testing data acquired from user 1 and user 2.

Users	SVM Acc	NB-Acc	DT-Acc	GB-Acc
User 1	84%	57	59	56
User 2	78	48	62	61
User 3	77.47	40.85	55	60.56
User 4	77.31	42	77.31	75.63
User 5	74.17	25.83	78.33	80
User 6	60	47.85	73.6	75
User 7	38.5	34.22	65.24	76
User 8	68	54.64	64	69
User 9	61.61	69.86	53.43	71.23

**Table 9:** Comparison of *F*-measure score obtained from user 1 and user 2.

Users	SVM-Acc	NB-Acc	DT-Acc	GB-Acc
User 1	84%	62	59	56
User 2	79	57	64	62
User 3	79	61.81	60.26	67.17
User 4	75.75	56	76.6	74
User 5	73.84	48.59	78.67	78
User 6	64	66.7	71.13	70.5
User 7	56	49.19	64.22	73.5
User 8	75	60.82	67.48	70
User 9	65.58	73	59.66	75.71

**Table 10:** Descriptive states of proposed features, with user 1 data.

Classifier name	User 1 data accuracy	User 2 data accuracy
SVM	13%	14%
Naive Bayes	31%	16%
Decision tree	39%	36%
Gradient boosted	32%	24%

## Data Availability

No data were used to support this study.
